# Application of Medical Imaging Based on Deep Learning in the Treatment of Lumbar Degenerative Diseases and Osteoporosis with Bone Cement Screws

**DOI:** 10.1155/2021/2638495

**Published:** 2021-10-11

**Authors:** Shengkai Mu, Jingxu Wang, Shuyi Gong

**Affiliations:** Shenyang Orthopedic Hospital, Shenyang, Liaoning 110044, China

## Abstract

**Objective:**

To explore the application value of magnetic resonance spectroscopy (MRS) and GSI-energy spectrum electronic computed tomography (CT) medical imaging based on the deep convolutional neural network (CNN) in the treatment of lumbar degenerative disease and osteoporosis.

**Methods:**

There were 56 cases of suspected lumbar degenerative disease and osteoporosis. A group of 56 subjects were examined using 1.5 TMR spectrum (MRS) and dual-energy X-ray absorptiometry (DXA) to collect the lumbar L3 vertebral body fat ratio (FF) and L1~4 vertebral bone mineral density (BMD) value. We divided the subjects into 2 groups with *T* value -2.5 as the critical point. Set *T* value > -2.5 as the negative group and *T* value ≤ -2.5 as the positive group. Pearson's method is used for FF-MRS and BMD correlation analyses. A group of all patients underwent GSI-energy spectrum CT scan, and X-ray bone mineral density (DXA) test results (bone density per unit area) were used as the gold standard to analyze the diagnosis of osteoporosis by the GSI-energy spectrum CT scan method value.

**Results:**

The differences in FF and BMD between the negative group and the positive group were statistically significant (*P* < 0.01), and there was a highly negative correlation between the average value of FF and BMD. 30 cases were diagnosed as osteoporosis by DXA. The accuracy of GSI-energy spectrum CT medical imaging in diagnosing osteoporosis is 89.30%. The GSI-energy spectrum CT diagnosis of osteoporosis and DXA examination results have good consistency.

**Conclusion:**

Based on the deep convolutional neural network (CNN) MRS technology, GSI-energy spectrum CT medical imaging is used in the clinical diagnosis and treatment of lumbar degenerative lesions and osteoporosis. It has a good advantage in assessing bone quality and has good consistency with DXA examination and has better application value high.

## 1. Introduction

Lumbar degenerative disease can cause spondylolisthesis, intervertebral disc herniation, lumbar spinal stenosis, etc. If it is combined with osteoporosis, it will undoubtedly accelerate the development of the disease. If some prognosis is not timely, segmental instability, small joint hyperplasia, and vertebral disc regression change, etc., is currently recognized as a problem that endangers global public health. At present, bone cement screws are often used for treatment, which can exert the advantages of high safety, easy operation, and less trauma, which is beneficial to the recovery and stabilization of limb function, and the prognosis effect is good [1]. Medical images can provide doctors with patient information to the maximum and have gradually become an important basis for doctors' diagnosis. Sometimes, they play a decisive role in doctors' diagnosis of diseases and the choice of treatment methods and methods.

In the past, the diagnosis of osteoporosis used DXA examination, energy spectrum CT, and magnetic resonance spectroscopy (MRS). The deep convolutional neural network (CNN) has excellent image classification capabilities and is applied to medical images. With the development of precision medical technology, medical image segmentation technology has become one of the researches focuses in the field of medical image processing. Based on this, this study explores the application value of diagnostic medical imaging based on deep learning in lumbar degenerative disease and osteoporosis.

## 2. Related Work

### 2.1. Inspection Technology

#### 2.1.1. DXA Inspection

According to recent research results, bone strength mainly depends on two aspects: BMD and bone quality. BMD refers to the combination of peak bone mass and bone loss, which can only reflect about 60% of the bone strength state; bone mass refers to bone metabolism, bone microstructure damage (including trabecular bone), and bone mineralization. The general term for bone biomechanics. DXA has been widely used to evaluate BMD due to its economy, simplicity, and low radiation, and WHO also recommends it as the “gold standard” for the diagnosis of OP [2]. However, DXA reflects the area density within the region and cannot effectively distinguish between cancellous bone and cortical bone, and the accuracy and sensitivity are poor.

#### 2.1.2. Magnetic Resonance Spectroscopy

Magnetic resonance spectroscopy (MRS) fat measurement technology uses chemical shifts to detect bone marrow water and adipose tissue and can measure its concentration. It can measure its concentration, analyze its biochemical composition and metabolic changes in vivo, and recognize the pathological changes from the molecular level. It is a new examination method for the diagnosis and prevention of osteoporosis.

The basis for the evaluation of osteoporosis by MRS technology: In the human body, bone marrow accounts for a relatively small proportion, but its main components, water and fat, are of great significance in the quantitative application of MRS bone marrow. Red bone marrow contains approximately 60% hematopoietic tissue (including water) and 40% adipose tissue; and yellow bone marrow contains more than 90% adipose tissue. When a person is born, there is almost red bone marrow in the bone marrow cavity. With age, the hematopoietic tissue and water in the bone marrow cavity gradually decrease, the trabecular bone becomes thinner and the gap expands, and the fat tissue continues to increase and fill it. The nature of the bone marrow is an important factor affecting bone quality. Bone marrow stem cell studies have confirmed that bone marrow adipocytes increase, compete, and inhibit the growth of osteoblasts to reduce them, which is an important mechanism leading to osteoporosis and fragility fractures. MRS can detect the water and fat components in the bone marrow and can quantitatively measure the fat fraction, thereby indirectly assessing the bone quality and opening up a new way for the early diagnosis and prevention of osteoporosis [3].

1H-MRS is the most commonly used technology in OP clinical and research. Earlier, Layer et al. confirmed the feasibility of 1H-MRS technology through in vivo bone marrow fat quantitative research. Recent domestic studies have also confirmed the accuracy and effectiveness of the application of 1H-MRS fat quantification technology. One of the most important indicators used by FF MRS fat quantification technology is also a hot research topic. FF stands for fat content. There are two commonly used definitions: one is the definition of signal intensity, that is, the ratio of fat signal intensity to the total signal intensity of water-fat; the other is to use the area under the peak definition, that is, the ratio of the area under the fat signal peak to the sum of the area under the water-fat peak, both of which are expressed as a percentage. Both definitions are used in the literature, but the definition of signal intensity is the most common [4]. It may be that the fat component is too complicated and the peak signal intensity is more representative. This study also adopted this definition.

#### 2.1.3. Energy Spectrum CT Scan

Energy spectrum CT can provide more accurate absolute CT values and can qualitatively separate and quantitatively determine and analyze substances. Its principle is mainly to calculate the spatial image by detecting the attenuation of X-rays and obtain the X-ray attenuation curve of the substance. The attenuation of each substance can be expressed by two “base substances.” The more common base substance pairs are iodine/water, hydroxyapatite (HAP)/water, and calcium/water, of which water and iodine are the two most commonly used base substances. Energy spectrum CT can quantitatively determine the content of calcium, HAP, and other minerals and fat in the vertebral body. Vertebral osteoporosis is mainly due to the decrease of bone mineral content in the vertebral body and the increase of bone marrow fat content. The representative of bone mineral is HAP, so the quantitative determination of HAP becomes the key to the diagnosis of osteoporosis. By measuring the quantitative parameters of energy spectrum CT, Dong Qiang and others found that the use of HAP/water as a base material is more accurate for the measured bone density, has a higher correlation with bone biomechanics, and can most accurately quantitatively evaluate bone strength.

In recent years, with the continuous development of spiral CT technology, GSI-energy spectrum CT medical imaging has been continuously used in the clinical diagnosis of osteoporosis because it can obtain images of water-based and calcium-based materials and has a certain value. Compared with conventional CT, GSI-energy spectrum CT can not only realize the diagnosis of density value and cell morphology but also analyze the imaging modes of multiple parameters. Its multiparameter imaging advantages greatly enrich the image information. Based on the temporal and spatial resolution of conventional CT, GSI-energy spectrum CT realizes imaging with energy resolution [5]. GSI-energy spectrum CT realizes the analysis of the chemical composition of the substance and the evaluation of the nature and function of the tissue through single-energy imaging, material separation technology, and the drawing of the energy spectrum curve, providing more information and reference [6].

### 2.2. Deep Convolutional Neural Network Image Segmentation Processing Technology

The convolutional neural network (CNN) is a type of feedforward neural network that contains convolutional calculations and has a deep structure. It is one of the representative algorithms of deep learning and the basis of many deep learning networks. Convolutional neural networks usually include an input layer, a convolutional layer, a pooling layer, and a fully connected layer, as shown in Figure 1.

Based on CNN, Long et al. proposed a fully connected network FCN, which solves the problem of input image quality degradation and low-resolution output caused by continuous convolution operations and pooling layers [7]. Inspired by FCN, Ronneberger et al. proposed the U-Net architecture, which is widely used in the field of medical imaging and later extended to a three-dimensional version to directly process three-dimensional images such as CT, as shown in Figure 2.

In the image classification task, CNN mainly performs a series of convolutional pooling operations on the image and then converts the image data into category probabilities through several fully connected layers for classification. In CNN, convolution is used to extract features, pooling is used to narrow the feature map to expand the convolution receptive field, and the fully connected layer reorganizes the features through the weight matrix. The results obtained through these operations are not easily affected by the feature and the position of the pixel itself in the image, so it has a good effect in the classification task. Medical image segmentation is of great significance in clinical diagnosis and treatment. For example, medical image segmentation can be used for 3D reconstruction of medical images, which is convenient for doctors to formulate surgical procedures, perform simulated operations, and quantify lesions [8].

Medical image segmentation, which is a computer-aided diagnosis technology applied in the medical field, can well help doctors complete the observation and analysis of medical images including magnetic resonance imaging, positron emission tomography, and computer tomography. Image segmentation is the area segmentation of the original image. The purpose of medical image segmentation is to obtain the anatomical structure of specific organs and tissues or to find regions of interest (ROI/VOI) by identifying contours and internal regions, such as lumbar degenerative lesions. Recently, deep learning technology has proven to be effective in segmenting tasks, and it is one of the common research topics in the field of deep learning applied medical imaging. The application methods of the deep convolutional neural network in medical image segmentation include transfer learning, hole convolution, and multiscale.

#### 2.2.1. Transfer Learning

CNN requires a large amount of labeled data for learning and modeling. However, in the medical field, especially medical image segmentation, it is very difficult to obtain a large number of labeled images, because it takes a lot of time for professionals to label, and the cost of labeling is very high. Therefore, transfer learning is suitable for the medical field. Migration learning uses neural networks pretrained with other data sets (the shallow network learns simple features, and the deep network learns complex features) and fine-tune the parameters of the network on the data set that needs to be segmented, thereby reducing the need for labeling data. Experiments show that using networks trained on similar data sets for migration learning has better data processing effects [9]. At the same time, the number of fine-tuning layers in migration learning should also be determined according to the similarity between the migration data set and the labeled data and the number of labeled data.

#### 2.2.2. Hole Convolution

In CNN, the pooling operation is usually used to reduce the size of the feature map and expand the receptive field, so that the network can learn more complex features, but each pooling operation will greatly reduce the image resolution, which is not good for pixel-level segmentation tasks. Therefore, the concept of hole convolution is introduced to replace the pooling operation to expand the receptive field, as shown in Figure 3 (the size of the convolution kernel is 3, the input stride is 2, and the output stride is 1) and Figure 2 (red in the figure). The point is the value in the original 3∗3 convolution kernel, and the remaining values are 0 [10–12]. Ordinary convolution takes an area with the same size as the convolution kernel each time, multiplies it pixel by pixel, and accumulates it as the convolution output of the center pixel of the area. The difference of hole convolution is that it adds the concept of rate of expansion (rate) to represent the distance between every 2 points in the convolution kernel. For example, when the expansion rate is 1, it is normal convolution, and when it is 2, it means that the two points in the convolution kernel are 1 pixel apart. The original 3∗3 convolution kernel will be equivalently expanded to 5∗5, which is the convolution kernel parameter shown in the red dot in Figure 2 (the nonred dots in the 5∗5 square are filled with 0). Equivalent to that in Figure 3, the input stride is 2 and the output stride is 1 convolution operation. This is equivalent to increasing the convolution kernel, that is, expanding the receptive field. This method is widely used in segmentation tasks.

#### 2.2.3. Multiscale

A number of studies have shown that the introduction of multiscale elements in the segmentation task can effectively improve the segmentation effect. Common methods are as follows.

*(1) Encoder-Decoder Model*. The encoding-decoding model is relatively common in the field of natural language processing and is also used in the field of image processing. The classic network U-Net in medical image segmentation uses the encoding-decoding model. U-Net first downsamples the image through a series of convolution pooling operations and then restores the image size through deconvolution to form a U-shaped structure, as shown in Figure 4. The convolution kernel of convolution and deconvolution requires parameter learning, and the original image of the same layer of convolution will be spliced as information supplement during each deconvolution.

*(2) Spatial Pyramid Pooling Method*. The established network structure often requires the input of fixed-size data, so that when processing pictures of different sizes, and the pictures must be cropped or scaled to a fixed size, causing some information to be lost. The spatial pyramid pooling method (spatial pyramid pooling (SPP)) can make the network adapt to any size of image input and, at the same time, use the classic feature extraction method of spatial pyramid to extract image features of different scales from the same image, so that the segmentation task can be further optimized [13]. SPP can also be combined with void convolution to form a new atrous spatial pyramid pooling (ASPP) method, which also has a good effect on segmentation tasks, as shown in Figure 5.

Another way to introduce multiscale elements is to downsample the input image from the beginning and then input the multiscale downsampling pictures into the network separately and combine to obtain the final segmentation result. This method is also used in medical image segmentation and has achieved better segmentation results than U-Net [14]. Taking a picture of 256∗256 pixels as the initial input data, 8x, 4x, and 2x downsampling was performed, respectively, and then the downsampling output results were input together with the original image into 4 segmentation networks; at the same time, the coarse-grained segmentation result is used as the input data and then input into the fine-grained segmentation network through supersampling. For example, perform 2x oversampling on the output result of 8 times downsampling and input the 4 times downsampling image together with the original image to obtain the 4 times downsampling segmentation result. In this way, the segmentation result of the original image is obtained by continuous refinement [15]. The 4 networks are also cyclically trained from coarse-grained to fine-grained one by one, as shown in Figure 6.

## 3. Materials and Methods

In order to improve the efficiency of diagnosis and reduce the amount of calculation, the diagnosis of lumbar degenerative disease and osteoporosis needs to detect the region of interest (ROI), that is, the lumbar region. The higher the detection accuracy, the maximum the removal of surrounding tissues and the preservation of the target area. The deep learning CNN algorithm is used to realize the detection function of the spine contour and the independent vertebra contour ROI area, and finally, the lumbar degenerative disease area is segmented through the contour overlap.

### 3.1. DXA Inspection and MRS Inspection

From April 2019 to September 2020, 56 cases (35 males and 21 females, age 40-80 years old) examined by dual-energy X-ray bone mineral density (DXA) were collected in our hospital. And the 1H-MRS examination was completed within 1 day to exclude endocrine, gastrointestinal, and kidney diseases that affect bone metabolism and absorption, various congenital and acquired abnormal bone metabolism diseases, multiple myeloma, and lumbar fractures. All subjects gave informed consent, and this study was approved by the ethics committee of our hospital.

The Lunar-Prodigy dual-energy X-ray bone densitometer from the American GE company was used to measure the patient's lumbar vertebrae 1 ~4 vertebral body and the femoral neck, intertrochanter, greater trochanter, and Ward's area of one hip [16]. Scanning conditions are as follows: tube voltage 140/100 kV and tube current 2.5 mA. Before the examination, instrument performance and quality control tests were performed, input of patient-related information was completed, and the patient was correctly positioned. The BMD value and *T* value of the abovementioned vertebral body were recorded. According to the recommended standards of the World Health Organization (WHO), *T* value = -2.5 is divided into 2 groups: >-2.5 is the negative group (normal or decreased bone mass) and ≤-2.5 is the positive group (OP).

We used the Philips Achieva1.5 T superconducting MR scanner (gradient field strength 27 mT/ms, effective switching rate 75 mT·m^−1^·ms^−1^) spine phased array surface coil. L3 vertebral body 1H-MRS scan was performed to exclude MR contraindications such as cardiac coronary stent implantation and claustrophobia. 1H-MRS scanning parameters are as follows: using single-point analysis spectrum (PRESS) for sagittal and transverse scanning, TR 3000 ms, TE 30 ms, reversal angle 90°, excitation times (NEX) 8 times, voxel (Voxel)20 mm × 20 mm × 15 mm, select the cancellous center of the vertebral body as the area of interest, and avoid the endplate cartilage and cortical bone. First, a saturation zone and parallel shimming around the area of interest were added, using unpressurized water MRS scanning [17]. Measure the water peak of the L3 cone at around 4.70 ppm and the lipid peak between 1.30 and 0.90 ppm. The research index fat ratio (FF) was collected, that is, the percentage of the relative signal intensity amplitude of fat to the total signal intensity amplitude (water and fat). The mathematical expression is

(1) $$\begin{array}{c} \text{FF}=\left[\frac{\text{Amapfat}}{\text{Ampfat}+\text{Anpwater}}\right]\times 100\%. \end{array}$$

The collected data is analyzed using the software that comes with the MR device.

The MRS scan was performed by an experienced technician, and the MRS images were read by two senior diagnostic imaging doctors [18]. If there is a difference in the results of the reading, an agreement is reached through consultation.

Using SPSS 19.0 statistical software, the FF value and BMD value measured by the MRS and DXA of the two groups were described by *x* ± *s* statistical parallel normality test, and the two groups conformed to the normal distribution. The *t*-test was used to analyze the correlation between the FF value and the BMD value by Pearson's method. The difference was statistically significant with *P* < 0.05.

### 3.2. DXA Inspection and Energy Spectrum CT Inspection

56 patients with suspected osteoporosis who were treated in our hospital from June 2017 to February 2019 were selected, including 22 males and 24 females; age 45-69 years, average (58.55 ± 5.05) years old, body weight 66~82 kg, and average body weight (76.00 ± 4.55) kg. This study was approved by the medical ethics committee of our hospital.

All patients undergo GSI-energy spectrum CT scan first and choose the German Siemens FLASH Hyun-speed two-photon CT machine. During the examination, keep the supine position and enter the bed with the foot first, and let the patient take a deep breath until the end of the scan to scan the patient's lumbar painful part. A tube voltage 80 kV, effective power supply 250 mAs, B tube 140 KV, effective current 125 mAs, open real-time dynamic exposure dose adjustment CARE Dose4D, collimator64 × 0.6 mm, pitch 0.7, speed 39.37 mm/cycle, rotation time 0.8 s/r, and at the same time, inject 300 mL of iohexol contrast agent (1.5 mL/kg) through the cubital vein at a rate of 3.0 ~ 3.5 mL/s, with a maximum of 100 mL of contrast agent. To scan to the lung nodules, the tube voltage and tube current should be adjusted to a low-dose 120 KV, 29 mAs. After the scan, the scanned image is transmitted to the VIA222266 workstation, the image data is processed by giveaway, and the calcium-water-based material image is obtained. The water-calcium density value of the three ROIs is measured at the vertebral cancellous level. Taking the average value, the determined ROI should include all the cancellous bone to the largest extent. The edge of the talar cortex is about 5 mm away from the bone island and venous plexus. The ROI is within 300 mm^2^ [19].

After the GSI-energy spectrum CT inspection is completed, DXA inspection is performed. For DXA inspection, GE Lunar Prodigy or iDXA model DXA scanner is selected, and the bone density of L1-4, femoral neck, and total hip is measured. Routine DXA scans of the lumbar spine and hips were performed. Bone density ROI includes L1-4, femoral neck, and total hip. The phantom scan was calibrated horizontally, using the European spine phantom (ESP-No. 145), and the patient's lesion was scanned approximately 10 times on the DXA machine. After each center completes the export of DXA data, it is uploaded to the data center, and the data is cleaned, checked, and corrected in a unified manner [20]. Divided by 5 years of age group, the average bone density of the patients at each site of the lesion in the sample was obtained, and the highest average bone density of the age group was selected as the peak bone density and the standard deviation, T = (bone density measurement − bone density peak value)/standard deviation, refer to the diagnostic criteria recommended by the World Health Organization in 1994, but each site *T* ≤ −2.5 is diagnosed as osteoporosis in this site of the patient.

Without knowing the DXA results at all, two radiologists with extensive experience will use a double-blind method to read the film together, and the diagnosis will be confirmed after discussion.

1. Diagnostic value: take the DXA test result as the “gold standard” for diagnosis, analyze the diagnostic value of GSI-energy spectrum CT medical imaging in the diagnosis of osteoporosis, with *a* for true positive, *d* for true negative, *c* for false positive, and *b* for False negative

(2) $$\begin{array}{c} \text{accuracy}=\frac{a+d}{a+b+c+d}\times 100\%,\\ \text{sensitivity}=\frac{a}{a+c}\times 100\%,\\ \text{specificity}=\frac{d}{b+d}\times 100\%\\ \text{positive predictive value}=\frac{a}{a+b}\times 100\%\\ \text{negative predictive value}=\frac{d}{c+d}\times 100\% \end{array}$$

(2) Consistency test: use Kappa to test consistency, and analyze the consistency of GSI-energy spectrum CT medical imaging to diagnose osteoporosis and DXA

We use SPSS 20.0 statistical software to analyze data and use Kappa to perform consistency test. When Kappa < 0.4, it indicates poor consistency; when 0.4 ≤ Kappa < 0.75, it indicates general consistency; when Kappa ≥ 0.75, it indicates good consistency, and *P* < 0.05 indicates that the difference is statistically significant.

## 4. Result Analysis

### 4.1. DXA Inspection and MRS Inspection Result Analysis

The FF-MRS and DXA bone mineral density test results of 56 subjects (24 cases in the negative group and 32 cases in the positive group) were collected for statistical analysis. After the *t*-test, the differences in FF and BMD between the negative group and the positive group were statistically analyzed. For academic significance (*P* < 0.01), see Table 1. The special cases are shown in Figures 7 and 8.

### 4.2. DXA Inspection and Energy Spectrum CT Inspection Result Analysis

For DXA results, among the selected 56 patients with suspected osteoporosis, 30 were diagnosed as osteoporosis by DXA.

In the comparison of the results of GSI-energy spectrum CT and MRI examination, the accuracy of GSI-energy spectrum CT scanning for osteoporosis is 89.30%, sensitivity is 86.67%, specificity is 92.31%, positive predictive value is 92.86%, and negative predictive value is 85.71%, see Table 2 for details.

In the consistency test, according to the Kappa consistency measurement, the GSI-energy spectrum CT diagnosis of osteoporosis and DXA test results are more consistent than the above. It is used in the clinical diagnosis of osteoporosis.

The accuracy, specificity, positive predictive value, sensitivity, and negative predictive value of GSI-energy spectrum CT medical imaging are not low, and the consistency with DXA examination is good, and the application value is high (Kappa = 0.786, *P* ≤ 0.001).

### 4.3. Bone Cement Screw Treatment

The patient was diagnosed with degenerative lumbar spine disease by X-ray and CT examination. The treatment method of bone cement screw are as follows: combined spinal-epidural anesthesia, prone position, posterior median surgery, and conventional tissue exposure, fix herringbone crest and joint For the face joints, lamina, and spinous process, and insert the needle at the apex of the lumbar herringbone ridge. After the guide needle is inserted, the direction and position of the positioning needle are appropriately adjusted under the guidance of the fluoroscopy machine. We further expand the nail channel (using a 5.5 mm opener), adjust the bone cement, pour it in at the early stage of the dough, and inject 1.5 mL bone cement into each nail channel. During the infusion, we pay attention to injecting and exiting. Bone cement push rod to ensure that the entire pedicle screw channel is completely filled, and then, all pedicle screws are inserted. Under the observation of the guiding machine, we check the dispersion in the vertebral body and prepare a disposable bone cement and place them separately; the 8 pedicle screws were adjusted to cement again. We pay attention to relieve the nerve compression, perform segmental decompression, remove the endplate cartilage and intervertebral disc nucleus pulposus, process the bone graft bed, and finally observe the position of the intervertebral fusion cage under guidance. If there is no abnormality, we suture the incision layer by layer, place a drainage tube, flush the wound, and cover with a sterile dressing. In postoperative treatment: the drainage tube can be removed within 48 hours after the operation, anti-infective drugs are used for three consecutive days, and bed rest is maintained for 14 days. The brace is protected for 1 to 2 months. Under the protection of the lumbar brace, the patient gets out of bed. After the operation, symptomatic treatments such as calcitonin or bisphosphonates, vitamin D, and calcium are needed.

After treatment, the Cobb angle of the fixed segment, the height of the adjacent upper intervertebral space, and the angle of the inferior endplate of the vertebral body were better than before treatment (*P* < 0.05), as shown in Figure 9.

## 5. Conclusion

DXA examination and energy spectrum CT examination result analysis showed that FF was closely related to BMD (*r* = −0.86, *P* < 0.01). According to research, bone density reduction is always accompanied by excessive accumulation of bone marrow adipose tissue. The bone marrow fat content of osteoporotic patients is significantly higher than that of healthy people of the same age. Li et al. also confirmed through experimental studies that increased bone marrow fat content is always accompanied by damage to the trabecular bone microstructure; Yeung et al. also made the same result and further pointed out that the unsaturated fatty acid index was significantly reduced during osteoporosis [21]. The index is obviously negatively correlated with fat content. Bone marrow fat accumulation and the imbalance between osteoblasts and fat cells are an important mechanism leading to osteoporosis. The diagnostic threshold of FF for osteoporosis is currently inconclusive. According to foreign reports, the range is about 58.2%-67.8%, which is basically in line with the results of this study 58.8%. Bone marrow fat is composed of multiple components, and it has been reported that there are no less than 20 types, but the specific relationship between each fat component and BMD is still unclear, and further research is still needed; secondly, the fat composition in the bone marrow may be different from the fat composition in other parts of the body. It shows that BMD is significantly negatively correlated with age and bone marrow FF but has no obvious correlation with gender, height, body weight, BMI, waist circumference, hip circumference, abdominal subcutaneous fat, and visceral fat. MRS technology has good advantages in assessing bone quality and can provide an effective auxiliary method for the assessment of primary osteoporosis.

The results of DXA examination and energy spectrum CT examination showed that the accuracy of GSI-energy spectrum CT scan for osteoporosis was 89.30%, the sensitivity was 86.67%, the specificity was 92.31%, the positive predictive value was 92.86%, and the negative predictive value was 85.71%; according to the Kappa consistency measurement, the GSI-energy spectrum CT diagnosis of osteoporosis and the DXA examination result have good consistency [20]. It shows that the sensitivity, accuracy, positive predictive value, specificity, and negative predictive value of GSI-energy spectrum CT medical imaging used in the clinical diagnosis of osteoporosis are at a high level, and the consistency with DXA examination is good. The application value is high. Scanning using GSI-energy spectrum CT medical imaging showed that long bones mainly showed thinning of the cortical bone, disordered or sparse bone trabeculae, stratification of bone, widening of joint space, surrounding bone degeneration, blurred trabecular structure, and other phenomena. The spine is deformed, the vertebral body is biconcave, the gap is widened, the bone trabecula is disordered, and the cartilage collapses, showing a fusiform or fishtail shape. In addition, the GSI-energy spectrum CT medical imaging uses single-tube dual energy to switch GSI in a short time. Due to its own material separation and material density quantitative measurement technology, it can obtain the GSI calcium-water density value of the cancellous bone of the vertebral body. Any object has a different X-ray energy absorption spectrum. When different base materials are combined, the X-ray attenuation will also change due to different X-ray absorption ratios. This process is called material separation [22]. When the matched base substance is the main component present in the tissue, measuring the value of the base substance can reflect the relative content of the substance in the tissue. In summary, in the clinical diagnosis of osteoporosis, the accuracy, specificity, positive predictive value, sensitivity, and negative predictive value of the GSI-energy spectrum CT medical imaging used in the clinical diagnosis of osteoporosis are not low and has better consistency with DXA inspection and higher application value.

Medical imaging is an important reference for doctors to make a diagnosis. Image segmentation helps doctors identify lesions and improve diagnosis efficiency. The deep learning method in medical image segmentation can reduce the influence of doctors' subjective factors and dig out hidden information from a large number of images. Deep learning does not require manual setting of parameters and automatic feature extraction without prior knowledge, which is convenient for doctors to use [23]. This can not only assist doctors in clinical diagnosis but also has important significance for medical big data research in the era of big data. In the future, in the context of further combining specific medical application scenarios with segmentation tasks, deep neural networks may become a major medical image segmentation method.

## Figures and Tables

**Figure 1:** The structure of the convolutional neural network.

**Figure 2:** Spine segmentation network structure for positioning+segmentation.

**Figure 3:** Hole convolution in one-dimensional state.

**Figure 4:** Classic U-Net structure.

**Figure 5:** ASSP method diagram.

**Figure 6:** Schematic diagram of cascade structure.

**Figure 7:** A 55-year-old male, osteoporotic MRS location map ((a) T2WI sagittal L3 vertebral body interest area and (b) T2WI transverse position L3 vertebral body interest area).

**Figure 8:** Male, 73 years old, osteoporosis ((a) MRS shows that the lipid peak at 1.30~0.90 ppm is significantly higher than the water peak at 4.70 ppm, FF = 59.3% and (b) BMD value measured by DXA = 0.758 g/cm^2^ and *T* value = -2.8).

**Figure 9:** After treatment with bone cement screws.

**Table 1:** Comparison of FF-MRS and BMD between the negative and positive groups.

Group	Number of cases	FF-MRS (%)	BMD (g/cm^2^)
Negative group	24	43.3 ± 0.3	1.22 ± 0.21
Positive group	32	73.2 ± 0.4	0.58 ± 0.45

**Table 2:** Comparison of GSI-energy spectrum CT scan results and DXA inspection results.

GSI-energy spectrum CT scan	DXA inspection results		Total
	Positive	Negative	
Positive	26	2	28
Negative	4	24	28
Total	30	26	56

## Data Availability

The image data used to support the findings of this study have been deposited in the VerSe 2019 data set (https://osf.io/nqjyw/).
